RETRACTED

# Identification of Histone Deacetylase 3 as a Biomarker for Tumor Recurrence Following Liver Transplantation in HBV-Associated Hepatocellular Carcinoma

**DOI:** 10.1371/journal.pone.0014460

**Published:** 2010-12-29

**Authors:** Li-Ming Wu, Zhe Yang, Lin Zhou, Feng Zhang, Hai-Yang Xie, Xiao-Wen Feng, Jian Wu, Shu-Sen Zheng

**Affiliations:** Key Lab of Combined Multi-Organ Transplantation, Key Lab of Organ Transplantation, Division of Hepatobiliary and Pancreatic Surgery, Department of Surgery, Ministry of Public Health, First Affiliated Hospital, Zhejiang University School of Medicine, Hangzhou, Zhejiang, China; Deutsches Krebsforschungszentrum, Germany

## Abstract

**Background:**

Recent studies have shown that high expression levels of class I histone deacetylases (HDACs) correlate with malignant phenotype and poor prognosis in some human tumors. However, the expression patterns and prognostic role of class I HDAC isoforms in hepatocellular carcinoma (HCC) remain unclear.

**Methodology/Principal Findings:**

The expression patterns and clinical significance of class I HDAC isoforms were assessed by immunohistochemistry in a cohort of 43 hepatitis B virus-associated HCC patients treated with liver transplantation. In addition, the effects of HDAC inhibition on HCC cell behavior were investigated by knockdown of the HDAC isoform with short interfering RNA. Class I HDACs were highly expressed in a subset of HCCs with positivity for HDAC1 in 51.2%, HDAC2 in 48.8%, and HDAC3 in 32.6% of cases. The expression levels of HDAC isoforms were significantly associated with the proliferation index of HCC. Kaplan-Meier curves showed that a high expression level of HDAC2 or HDAC3 implicated significantly reduced recurrence-free survival. Cox proportional hazards model analysis revealed HDAC3 overexpression was an unfavorable independent prognostic factor (P = 0.002; HR 3.907). *In vitro*, inhibition of HDAC2 and HDAC3, but not HDAC1, suppressed proliferation and the invasiveness of liver cancer cells.

**Conclusions/Significance:**

Our findings demonstrate that HDAC3 plays a significant role in regulating tumor cell proliferation and invasion, and it could be served as a candidate biomarker for predicting the recurrence of hepatitis B virus-associated HCC following liver transplantation and a potential therapeutic target.

## Introduction

Hepatocellular carcinoma (HCC) is the most common primary malignant tumor in liver. It ranks fifth in incidence and fourth in mortality rate in overall tumors [1], [2]. China is one of the highest prevalent areas of HCC, mainly because chronic hepatitis B carriers account for more than 10% of the Chinese population [3]. The prognosis of patients with HCC is generally poor, even after surgery or chemotherapy. Liver transplantation (LT) offers a potential curative option for patients with small HCC. However, frequent recurrence or metastasis after transplantation remains the main obstacle for long-term survival [4]. Therefore, elucidating the molecular mechanism of HCC recurrence is vital for the development of more effective therapeutic strategies.

RETRACTED

Evidence has shown that modifications of acetylation play an important role in tumor progression and metastasis [5], [6]. Histone deacetylases (HDACs) are known to be one of the major enzymes that change the nucleosomal conformation of tumor cells via post-translational deacetylation of the core histones. Therefore, aberrant activation of HDACs leads to transcriptional repression of diverse genes mainly involved in the regulation of behavior of tumor cells such as proliferation, differentiation, angiogenesis and invasion, as well as migration and metastasis [7], [8].

So far, eighteen HDAC isoforms, grouped into four classes, have been described in humans [9]. Among them, the best characterized and probably biologically most relevant HDACs were class I isoforms HDAC1, HDAC2 and HDAC3. The expression patterns of HDAC1, HDAC2 and HDAC3 have been evaluated in different types of cancers, including gastric cancer [10], colorectal cancer [11], prostate cancer [12], breast cancer [13], renal cell cancer [14], and ovarian and endometrial carcinomas [15]. Elevated expression of class I HDAC has been shown to be an unfavorable independent prognostic factor in some of these tumor entities [16]. However, little is known on the expression pattern and biologic function of a single HDAC isoform in HCC, especially in HCC treated with LT.

Recently, a new group of chemotherapeutics called histone deacetylase inhibitors (HDIs) have emerged. HDIs, such as valproic acid (VPA) and suberoylanilide hydroxamic acid (SAHA) target the HDAC enzyme family. VPA and SAHA, inhibiting class I and class II HDACs, causes growth arrest, differentiation and/or apoptosis of tumor cells, and considered to be potential substances for the treatment of malignant solid human tumors in the near future [17], [18]. However, the contribution of specific HDAC isoforms to the tumor progression, invasion and metastasis is still unclear.

In the present study, we investigated the expression patterns of HDAC1, HDAC2 and HDAC3 in HCC patients following LT and analyzed their relationship to the clinical phenotype, using a clinically well-characterized cohort of HCC patients treated with LT. Meanwhile, the functions of specific class I HDAC isoforms in liver cancer cells were also characterized.

RETRACTED

## Methods

### Ethics statement

The study protocol was approved by the Institutional Review Board of Key Lab of Combined Multi-organ Transplantation, Ministry of Public Health. Informed written consent was obtained according to the Declaration of Helsinki.

### Study population and tissue samples

Forty-three HCC patients treated with LT during 2003 and 2005 in our hospital (First Affiliated Hospital, Zhejiang University School of Medicine, Zhejiang, China) were enrolled in this study. The eligibility criteria for the patients studied are as follows: (a) HCC diagnosed either before or after transplantation (as an incidental finding), which was confirmed by histopathological examination; (b) the patients were Han Chinese; (c) complete clinical and laboratory data such as portal vein tumor thrombi (PVTT), preoperative alpha-fetoprotein(AFP) level, histopathologic grading, tumor size, and tumor number were available before operation and during follow-up; (d) all patients were HBV-positive (HBsAg+) and none of them were hepatitis C virus (HCV)-positive; (e) none of the patients received preoperative adjuvant antineoplastic therapy; and (f) absence of de novo HCC nodules occurring in the transplanted liver. Follow-up data were obtained after LT for all 43 patients. The follow-up course and diagnostic criteria of recurrence has been described previously [19]. The distribution of the clinicopathologic data in the study cohort is given in Supplementary Table S1.

### Cell lines

Liver cancer cell lines SMMC-7721 and HepG2, as well as the metastasis-capable human HCC cell lines MHCC97L (intermediate metastatic capability) and HCCLM3 (the most metastatic capability) were purchased from American Type Culture Collection (Manassas, VA) and Shanghai Institute of Cell Biology (Shanghai, China).All of the cell lines were maintained in the recommended culture conditions and incubated at 37°C in a humidified environment containing 5% CO_2_.

### Immunohistochemistry

Tissue sections of 4-µm thickness were stained with monoclonal mouse HDAC1 antibody (1∶80; Abcam, Cambridge, UK), monoclonal mouse HDAC2 antibody (1∶5000; Abcam), monoclonal rabbit HDAC3 antibody (1∶80; Abcam) and monoclonal mouse Ki-67 antibody (1∶100; Zhongshan, Beijing, China). The immunohistochemistry procedure has been described previously [20]. Nuclear staining of HDAC1, HDAC2 and HDAC3 was scored using a semi-quantitative immunoreactivity scoring (IRS) system [11]. The immunostained sections were independently evaluated by two pathologists who were blind to the clinical data. Cases with an IRS from 0 to 6 were defined as HDAC negative, while cases with an IRS higher than 6 were defined as HDAC positive. The Ki-67 index was determined by counting Ki-67-positive nuclei per 100 tumor cells in a representative tumor section.

RETRACTED

### HDIs treatment and RNA interference

Cells were seeded into plates with a density of 5×10^4^/mL, cultured for 24 hours, then treated with SAHA (Alexis Biochemicals, San Diego, CA) and VPA (Sigma, St.Louis, MO) at a concentration of 2.5 µM and 2 mM, respectively. After evaluating the effects of chemical HDI, we analyzed the specific function of Class I HDAC isoforms in liver cancer cells. Select validated short interfering RNA (siRNA) duplexes (Ambion, Austin, TX) were used to detect RNA interference-mediated down-regulation of HDAC1, 2, 3, and a nonsilencing siRNA was used as negative control. After 24 hours, cells were transfected with 33 nM siRNA using Lipofectamine2000 transfection reagent (Invitrogen, Carlsbad, CA) according to the manufacturer's instructions. The efficacy of transfection was checked by Reverse Transcription Polymerase Chain Reaction (RT-PCR) after 48 hours of incubation.

### Cell viability assay and cell cycle analysis

Following treatment with HDIs or siRNA for 72 hours, cell viability was detected using a cell counting kit-8 (Dojindo Laboratories, Kumamoto, Japan) according to the manufacturer's instructions. Cells were then incubated at 37°C for another 2 hours and measured at 450 nm and 630 nm. The experiment was repeated three times.

To detect the cell cycle alterations, cells were treated with HDAC1, 2, 3 siRNA, VPA and SAHA as described above. Cells were then harvested and stained with DNA PREP kit (Beckman Coulter, Fullerton, CA). The percentage of cells in sub G1, G0/G1, S, and G2/M phase was quantified using flow cytometry analysis according to the manufacturer's instructions (CYTOMICS FC 500, Beckman Coulter). The extent of apoptosis was assessed by the proportion of cells giving fluorescence in the hypodiploid sub G1 peak of the cell cycle. Analysis of cell cycle data was done with MULTICYCLE analysis software. All experiments were done in triplicates.

### Cell invasion assay

Cell invasion analysis was performed using a Transwell (Millipore, Billerica, MA) based method. Seventy-two hours after RNA interference, 200 µL of 0.8×10^5^ cells were applied to the upper compartment of the matrigel (BD Bioscience, San Jose, CA) coated filters, while the lower compartment was filled with Dulbecco's modified Eagle's medium supplemented with 15% fetal bovine serum. After 48 hours, migrated cells on the bottom surface were fixed with methanol and stained with 0.1% Crystal Violet. The invading cells were examined, counted, and photographed using digital microscopy (×200). Four fields were counted per filter in each group.

RETRACTED

### Semiquantitative reverse-transcription polymerase chain reaction

Total RNA was extracted from all the cell lines using TRIZOL (Invitrogen, Carlsbad, CA). Two micrograms of total RNA was used for cDNA synthesis in each reaction. PCR were performed for HDAC1, HDAC2, HDAC3, and β-actin. The primers are listed on Supplementary Table S2. Relative gel band intensities of the products were measured by Kodak digital science image system (Kodak, Rochester, NY).

### Statistical analysis

The association between Class I HDAC expression and clinicopathological variables was assessed by using either the Pearson's chi-square test or two sided Fisher's exact test, as appropriate. The correlation of Class I HDAC expression and tumor recurrence was evaluated according to Kaplan-Meier estimates. Cox regression was applied to assess variables significantly associated to recurrence in the univariate analysis. The detailed statistical tests used in the study are given in Results, and in the Tables and Figure legends. Statistical analysis was performed with SPSS 15.0 and GraphPad Prism 5.0. All tests were two tailed and P<0.05 was considered statistically significant.

## Results

### Expression patterns of Class I HDAC isoforms in HCC

High expression levels of all three HDAC isoforms (HDAC1, HDAC2 and HDAC3) in HCC nuclear were observed. In 43 cases, 22 (51.2%), 21 (48.8%) and 14 (32.6%) cases were positive for HDAC1, HDAC2 and HDAC3, respectively (Supplementary Table S1; Figure 1A). In some cases, additional cytoplasmic positivity was observed in a minority of tumor cells. Furthermore, all of the three HDAC isoforms were detectable in the nuclei of the bile duct. Stromal cells of HCC also displayed weak to moderate nuclear positivity for all of the three HDAC isoforms, which might be due to positive staining in fibroblasts and infiltrating inflammatory cells.

**Figure 1:** The role of class I HDAC expression in HCC patients receiving liver transplantation. (A) Representative HDAC1-positive (a,b), HDAC2-positive(c,d) and HDAC3-positive(e,f) samples are shown at 100× (a,c,e) and 400× magnification (b,d,f). HDAC negative (IRS from 0 to 6) and HDAC positive (IRS higher than 6). (B) Kaplan-Meier curves estimates the recurrence-free survival rates according to expression patterns of HDAC1, 2, 3, and combined HDAC expression in the cohort.

### Correlation of Class I HDAC isoforms expression with clinicopathologic variables and cell proliferation

The association of the expression levels of HDAC isoform with clinicopathologic variables were further analyzed. Resultantly, the expression level of HDAC1 and HDAC2 was only associated with Ki-67 index (HDAC1, P = 0.021; HDAC2, P = 0.044), while HDAC3 was associated with Ki-67 index (P = 0.001) and tumor size (P = 0.005) (Supplementary Table S1). In addition, when the patients were grouped according to their overall class I HDAC expression pattern (all three isoforms negative versus one or two isoforms positive versus all three isoforms positive), positive expression of all three isoforms was associated with enhanced Ki-67 index as a surrogate marker of proliferation (P<0.001, one way ANOVA) and tumor size >5 cm (P = 0.033, χ^2^ test for trends; Supplementary Table S1).

RETRACTED

### Correlation of Class I HDAC isoforms expression and recurrence

To determine whether changes in class I HDAC expression were relevant to the recurrence of HCC patients treated with LT, univariate and multivariate survival analysis were performed. Patients with a high expression level of HDAC2 or HDAC3 were prone to earlier recurrence of HCC according to Kaplan-Meier estimates (Table 1, Figure 1B). Furthermore, we observed that the difference was pronounced when the HDAC all positive expression group was compared with HDAC all negative expression group (P = 0.015; Figure 1B). Univariate analysis also revealed that the clinicopathological variables could provide significant predictive values for recurrence including PVTT (P = 0.024), preoperative AFP level (P = 0.004), tumor size (P = 0.004), and tumor number (P = 0.017) (Table 1). These results were consistent with those previous reports in terms of clinical histological features [19], [21], which suggests that the selected samples in this study reflect the characteristics of LT patients in the Chinese population. Multivariate analysis further revealed that HDAC3 expression level was a novel independent factor (P = 0.002; hazard ratio 3.907) for predicting recurrence-free survival (Table 2).

**Table 1:** Influence of HDAC isoform expression and clinicopathologic variables on HCC recurrence.

Variables	Grading	Recur		P*
		Negative	Positive	
Age(Years)	≤50	9	13	0.278
	>50	12	9	
Gender	Female	1	1	0.788
	Male	20	21	
PVTT	Negative	16	10	0.024
	Positive	5	12	
Preoperative AFP level (ng/ml)	≤400	15	8	0.004
	>400	6	14	
Histopathologic grading	Well+moderate	17	16	0.884
	Poor	4	6	
Tumor size (cm)	≤5	12	4	0.004
	>5	9	18	
Tumor number	Single	12	5	0.017
	Multiple	9	17	
HDAC1	Negative	13	8	0.228
	Positive	8	14	
HDAC2	Negative	16	6	0.010
	Positive	5	16	
HDAC3	Negative	19	10	0.001
	Positive	2	12	
HDAC groups	All negative	10	5	0.015
	Partially positive	10	6	
	All positive	1	11	

*Log-rank test.

**Table 2:** Multivariate Cox regression analysis of variables related to tumor recurrence at univariate analysis.

Variable	HR(95% CI)	P
AFP		
<400 ng/ml	1.000	
>400 ng/ml	3.520(1.441–8.598)	0.006
HDAC3		
Negative	1.000	
Positive	3.907(1.623–9.403)	0.002

Abbreviations: HR, risk ratio; 95% CI, 95% confidence interval.

RETRACTED

### Inhibition of cell proliferation and cell cycle alterations by treatment with VPA and SAHA

In vitro, we tested the effects of chemical HDI on liver cancer cells (SMMC-7721, HepG2, MHCC97L and HCCLM3). Treatment of liver cancer cells with SAHA (maximum dose 5 µM) and VPA (maximum dose 4 mM) both revealed a significant dose-dependent reduction in cell number after 72 hours (Figure 2A).

**Figure 2:** Antiproliferative effects of chemical HDAC inhibitors and selective HDAC1, 2, 3 silencing in HCC cells. (A) Treatment with either VPA or SAHA led to a significant dose-dependent reduction of HCC cell numbers after 72 h. (B) Effective silencing of HDAC1, 2, 3 mRNA in HepG2 after siRNA treatment for 48 hours. (C) Selective knockdown of HDAC3 and HDAC2 led to reduction of HepG2 cell numbers after 72 hours (**P<0.01, Student *t* test).

In addition, treatment of liver cancer cell lines with VPA (2 mM, 48 or 72 hours) resulted in an accumulation of cells in G0-G1 phase of the cell cycle. In contrast, treatment with SAHA (2.5 µM, 48 or 72 hours) led to an accumulation of cells in the G2-M phase (Figure 3A; Supplementary Table S3). Meanwhile, treatment with SAHA, and to a lesser extent of VPA, led to a significant induction of apoptosis of liver cancer cells in a time-dependent manner.

**Figure 3:** Apoptosis-inducing and cellcycle alteration effects of HDIs and selective HDAC siRNA silencing in HCC. (A) Flow cytometric analysis of apoptosis and cell cycle in 4 HCC cell lines after the treatment with the DMSO vehicle or the indicated concentrations of VPA and SAHA for 24, 48, or 72 hours. (B) Apoptosis and cellcycle alterations in HepG2 after selective silencing of HDAC1, 2, 3 for 48 hours.

### Inhibition of cell proliferation and cell cycle alterations by specific silencing Class I HDAC isoforms

To further understand the function of Class I HDAC isoforms in liver cancer cells, specific class I HDAC isoforms were knockdowned by siRNA in HepG2 cell. The data showed that treatment with selective siRNA led to a specific reduction of mRNA expression of the HDAC isoforms (Figure 2B). In addition, selective knockdown of HDAC1, HDAC2 and HDAC3 resulted in a reduction of 5.3%, 19.7% and 29.7% in cell number, respectively. However, only the difference for HDAC2 and HDAC3 was statistically significant (P<0.05; Figure 2C).

Similarly, knockdown of HDAC2 and HDAC3 in HepG2 resulted in an accumulation of cells in G2-M and a reduction of cells in the S phase (Figure 3B; Supplementary Table S3), while specific knockdown of HDAC1 showed no obvious effect on the cell cycle after 48 hours. No significant induction of apoptosis in HepG2 was observed after treatment with isoform-specific siRNA in the present study (Figure 3B).

RETRACTED

### Inhibition of invasion of HCC cells by specific silencing Class I HDAC isoforms

As shown in Figure 4C, the inhibitory efficiency of siRNAs for gene transcription was significant in high-metastasic potential HCCLM3 cells. To determine whether knockdown of specific HDAC isoform had a crucial role in cell invasion, we performed an *in vitro* cell invasion assay. The result showed that the average number of invaded cells transfected with HDAC2 or HDAC3 siRNA significantly decreased when compared to those with negative control siRNA (Figure 4A, B). This indicates that the invasive potential of HCCLM3 cells was suppressed after transfection of HDAC2 and HDAC3 siRNA. In line with the hypothesis that HDAC2 and HDAC3 may be important contributors to the invasion of tumor cells, the expression levels of HDAC2 and HDAC3 influenced the metastatic behavior of the HCCLM3 cell line.

**Figure 4:** Alteration of class I HDAC isoform levels in HCCLM3 cells changes its invasiveness in vitro. (A) Selective knockdown of HDAC3 and HDAC2 led to reduced invasiveness of HCCLM3 (**P<0.01, Student *t* test). (B) Representative images of invasiveness of HCCLM3 cells transfected with negative siRNA (a) or siRNA against HDAC1(b), HDAC2(c), and HDAC3 (d). The transwell invasion assay showed that HCCLM3 cells transfected with siRNA against HDAC2,3 displayed a markedly decreased invasiveness behavior, as indicated by a significant decrease in the average number of cells invaded through the matrigel in comparison with the control siRNA. (C) Effective silencing of HDAC1, 2, 3 mRNA in HCCLM3 after siRNA treatment for 48 hours.

## Discussion

In the present study, class I HDAC isoforms (HDAC1, HDAC2, and HDAC3) were highly expressed in a panel of HCC cases. High expression levels of HDAC2 and HDAC3 were associated with significantly reduced recurrence-free survival, with HDAC3 being an independent prognostic factor in this cohort. In addition, respective silencing of HDAC2 and HDAC3 suppressed proliferation and the invasiveness of HCC cell lines *in vitro*. To our knowledge, this is the first detailed systematic investigation of the expression pattern and the role of these three proteins in HCC.

Increasing numbers of studies suggest that expression of class I HDACs is associated with clinicopathological parameters or tumor prognosis in several types of cancer [10]–[12]. In a study of prostate cancer, Weichert et al [12] demonstrated that high expression levels of class I HDACs correlated with higher proliferative fractions (measured by Ki-67). Similar results were also observed in the present study. Expression of HDAC1 (P = 0.021), HDAC2(P = 0.044) and HDAC3 (P = 0.001) were all associated with the Ki-67 index of liver cancer cells (Supplementary Table S1). These data suggest that high HDAC activity leads to enhanced tumor cell activity. Based on these findings, we speculated that the expression level of class I HDACs might be associated with tumor recurrence in LT patients for HCC. We found that expression of HDAC3 was an independent factor influencing the risk of recurrence in HCC patients following LT, which is in line with the *in vitro* results of proliferation, cell cycle, and invasion (Figure 2, Figure 4). These data suggest HDAC3 expression may serve as a novel candidate prognosticator for HCC treated with LT, although the finding ought to be verified in a larger prospective study.

RETRACTED

On the other hand, the functional studies of liver cell lines with siRNAs targeting class I HDACs showed no obvious difference between the knockdown of HDAC2 or HADC3 expression in the amount of viable cells, as well as in the amount of invasive cells. Some recent studies also have demonstrated that high HDAC2 expression is associated with shortened relapse-free survival time or overall survival time in different types of cancer [10], [12]. However, in the present study, only HDAC3, not HDAC2 showed an independent specific role in predicting recurrence of HCC following liver transplantation. This discrepancy might be due to the small sample size, which is similar to most of the cohorts previously investigated.

In addition, elevated HDAC1 expression showed no influence on the risk of recurrent HCC after LT in the present study, which is contrast to the previous study for 47 Japanese patients with surgically resected HCC [22]. Possible explanations for the discrepancy in these results include difference in the studied cohorts, including variation in the genetic and etiology backgrounds of the patients. Despite the important role of HDAC3 in tumor recurrence and its predictive implications, this study should be viewed as hypothesis generating, to be followed by larger prospective and multiethnic studies to confirm our findings.

Previous studies *in vitro* have suggested that chemical HDI (VPA and SAHA) could reduce cell proliferation, induce cell cycle arrest and apoptosis of several liver cancer cell lines [23]–[25]. Obviously, our results confirmed these effects in a range of liver cancer cells. However, current data on the cellular effects of a specific HDAC isoform knockdown in liver cancer is unclear. To clarify whether the effects of VPA and SAHA inhibition could be contributed to an inhibitory effect on one specific class I HDAC isoform, we investigated the effect of HDAC1, HDAC2, or HDAC3 on the proliferation, cell cycle, apoptosis and invasion of HCC cells by means of RNA silencing. Consistent with the above mentioned results *in vivo* (Supplementary Table S1), we found that silencing of HDAC2 or HDAC3 significantly reduced cell numbers and induced cell cycle arrest in HepG2 cells, suggesting that selected class I HDAC isoforms may play an important role in regulating tumor cell proliferation. Supporting our results, a previously published study demonstrated similar effects in colon cancer cell lines [26]. In addition, similar to the results of Spurling et al [27] in SW480 cells, the invasive capacity of HCCLM3 cells was significantly reduced after HDAC2 or HDAC3 knockdown, indicating that these two isoforms are involved in the invasion and metastasis processes of HCC cells. In the preset study, we chose HCCLM3 as the representative HCC cell line to analyze the invasiveness influence of HDACs, therefore, the observed results and mechanisms might be limited to this cell line. We can get more detailed data by evaluating additional metastatic potential cell lines, such as MHCC97L and MHCC97H. Taken together, these findings suggest that HDAC2 and HDAC3, especially HDAC3, may be important regulators for the proliferation and invasion of HCC cells, which at least partly explained the mechanism of tumor recurrence *in vivo*, and could be possible targets for suppressing tumor viability.

RETRACTED

Our findings confirm the cellular biological basis that Class I HDACs exert a tumor-promoter effect in HCC through the induction of cell proliferation, invasion and metastasis. HCC cell proliferation and invasion involves in multiple steps and required alterations of a variety of tumor related genes, such as CDKN1A, E-cadherin, T-cadherin, DACT3, and MMP-2 [26], [28]–[30]. To comprehensively understand the exact molecular mechanism of the class I HDACs regulation, gene expression microarray analysis involving tumor proliferation and metastasis pathways, should be conducted.

The HBV contribution for the current findings should be highlighted in the present study. Recently, the induction of HDAC1 by HBV X protein has been reported [31], [32], and could act as a confounding factor. In the present study, the studied population almost unavoidably consisted of patients with hepatitis B virus-associated HCC because of the special situation in China. The analysis of HDACs expression in liver tissue of HCC patients with other etiological backgrounds might be very useful to ascertain the real predictive value of HDAC3 for HCC recurrence.

RETRACTED

In summary, our results demonstrated the important role of class I HDACs, especially HDAC3, in liver cancer biology. Patients showing elevated HDAC3 expression had a significant negative prognostic impact in terms of recurrence-free survival, which indicates the potential use of this molecular marker to predict patient risk of recurrence after LT. More importantly, the prognostic impact of HDACs, together with our observation of the proposed interactions of HDAC isoforms with tumor cell proliferation and invasion, strongly suggests targeting class I HDACs might be an effective therapeutic strategy for HCC patients after LT.

## Supporting Information

Table S1 Overall expression of class I HDAC isoforms in HCC treated with LT as well as the distribution of clinicopathologic data in this study cohort.
(0.10 MB DOC)

Table S2 Primers sequences for RT-PCR analysis of related genes described in this paper.
(0.03 MB DOC)

Table S3 Distribution of HepG2 cells in different phases of cell cycle after treatment with VPA, SAHA and HDAC1, HDAC2 as well as HDAC3 siRNA after 48 hours. Experiments were performed in triplicates.
(0.03 MB DOC)
